# Vibrational, electronic, spectroscopic properties, and NBO analysis of p-xylene, 3,6-difluoro-p-xylene, 3,6-dichloro-p-xylene and 3,6-dibromo-pxylene: DFT study

**DOI:** 10.1016/j.heliyon.2020.e05783

**Published:** 2020-12-23

**Authors:** Emmanuel A. Bisong, Hitler Louis, Tomsmith O. Unimuke, Joseph O. Odey, Emmanuel I. Ubana, Moses M. Edim, Fidelis Timothy Tizhe, John A. Agwupuye, Patrick M. Utsu

**Affiliations:** a Department of Pure and Applied Chemistry, Faculty of Physical Sciences, University of Calabar, Calabar, Cross River State, Nigeria; b Computational Quantum Chemistry Research Group, Department of Pure and Applied Chemistry, Faculty of Physical Sciences, University of Calabar, Calabar, Cross River State, Nigeria; c Department of Textile and Polymer Engineering, Ahmadu Bello University, Zaria, Nigeria; d Institute of Chemistry, Chinese Academy of Sciences, 10900 Beijing, China; e Department of Chemistry, Cross River University of Technology, Calabar, Calabar, Cross River State, Nigeria

**Keywords:** DFT, NBO, Frequency, Spectroscopy, PX, DFPX, DCPX, DBPX

## Abstract

This study explains the vibration and interaction of p-xylene and effect of three elements (fluorine, chlorine and bromine) of the halogen family substitution on it. Basic chemistry of four, compounds p-xylene (PX); 3,6-diflouro-p-xylene (DFPX); 3,6-dichloro-p-xylene (DCPX) and 3,6-dibromo-p-xylene (DBPX) has been explained extensively using theoretical approach. Vibrational energy distribution analysis (VEDA) software was used to study the potential energy distribution (PED) analysis, bond length, bond angles and dihedral angles of PX, DFPX, DCPX, DBPX after optimization with GAUSSIAN 09 software. The trend in chemical reactivity and stability of the studied compounds was observed to show increasing stability and decreasing reactivity moving from DBPX, DCPX, DFPX to PX and this was obtained from the calculated highest occupied molecular orbital (HOMO) and lowest unoccupied molecular orbital (LUMO) values. Our results show that PX is the best electron donor (best nucleophile) while DBPX is the best electron acceptor (the best electrophile). We also observed that the substituted halogen increases the value of the bond angles but the effect is reduced as the size of the halogen increases. The maximum intensity and the frequency value for the maximum intensity of the different compounds was determined using the VEDA 04 software**.** From our natural bond orbital (NBO) 7.0 program analysis, the studied compounds are said to show biological activities as well as the intramolecular hyperconjugative interactions responsible for stabilizing the compounds. The NBO results also revealed that the non-bonding interaction existing between the lone pair electron on the halogen atoms and the aromatic ring increases the stability of the halogen substituted para-xylene molecules. Multiwfn: A Multifunctional Wavefunction Analyzer was used for the spectroscopic plots.

## 1 Introduction

Xylene is an aromatic compound that has methyl groups substituted on benzene ring. The substitution occurs at two positions in the ring. Depending on the positions of methyl groups in the benzene ring, xylene could be classified into ortho xylene (o-xylene), meta xylene (m-xylene) and para xylene (p-xylene) [1, 2, 3]. Xylene is found to be predominant in the carbonization of coal producing coke fuel. It is the major precursor in terephthalic acid and dimethyl terephthalate which are being utilized in polyethylene terephthalate (PET) production and related derivatives of which p-xylene is the building block of PET. [4, 5] Scientific studies on p-xylene have been reported by many researchers. C. Venkatesh *et. al.* reported structural, electronic and optical properties of 2,5-dichloro-p-xylene using experimental and DFT approaches [1]. Manzoor, M. studied chemical properties and anticancer activity of tetra bromo-p-xylene [6]. So far, they have been no report on *in silico* study on halogen effect of p-xylene in terms of quantum chemical descriptors, natural bond orbital (NBO) and spectroscopic study using DFT. Hence, the need for this study. We are inquisitive to know how halogen affect p-xylene, we looked at quantum chemical descriptors, NBO and spectroscopic properties of p-xylene as well as 3,6-di-(flouro, chloro and bromo) p-xylene. We observed an interesting trend in chemical reactivity and stability of the studied compounds to show increasing stability and decreasing reactivity moving from DBPX, DCPX, DFPX to PX and this was obtained from the calculated highest occupied molecular orbital (HOMO) and lowest unoccupied molecular orbital (LUMO) values. Our results show that PX is the best electron donor (best nucleophile) while DBPX is the best electron acceptor (the best electrophile). The DFT method using the hybrid exchange correlation functional B3LYP have been employed in this research due to its effectiveness and accuracy in the investigation of conjugated systems or lone pair containing species and vast application in various researches reported in literature.

## 2 Computational details

To explain the chemistry of PX, DFPX, DCPX and DBPX, 2,5 DCPX was obtained from literature [1] through which others were designed and the calculation was done using GAUSSIAN 09W and GAUSS VIEW 0.6 [7, 8], Vibrational Energy Distribution Analysis (VEDA) 4 softwares [9] and Natural Bond Orbital (NBO) 7.0 program [10]. GAUSSIAN 09W was used for optimization. The geometry optimization was performed using density functional theory (DFT) with Becke's three parameter exchange-functional combined with corrected correlation Lee, Yang and Parr functional (B3LYP) methods using 6-311+G(d,p) basis and spectroscopic studies. Natural bond orbital (NBO) 7.0 program was used to study inter molecular charge transfer (ICT) as well as stability of p-xylene (PX), 3,6-diflouro-p-xylene (DFPX), 3,6-dichloro-p-xylene (DCPX) and 3,6-dibromo-p-xylene (DBPX), while VEDA 04 was used to study the vibrational properties of the compounds. Multiwfn: A Multifunctional Wavefunction Analyzer was used for the spectroscopic plots [11].

## 3 Results and discussion

### 3.1 Geometrical parameters

The values of bond length, bond angle and the dihedral angle were calculated using GAUSSIAN-09W and vibrational energy distribution analysis (VEDA) softwares. Tables 1, 2, and 3 compare the theoretically calculated bond lengths, bond angles, and dihedral angles of PX, DFPX, DCPX, and DBPX. It is evident from the values obtained that the substituted carbons have large bond lengths when compared to the halogen and as the size of the halogen increases the value of the bond length also increase. The first statement could be due to the positive inductive effect (+I) of the methyl group, and negative inductive effect (-I) of the halogen and also the resonance effect of the phenyl ring. The + I effect of the methyl group confers on it an electron donor and so it pushes electrons into the benzene ring. The negative inductive effect of the halogen and resonance effect of the phenyl ring comes together to pull the electrons towards themselves. The net result is that the bond length of carbon substituted by methyl group is larger compared to the bond length of carbon substituted by halogen [12]. The second statement is explained based on the fact that as the size of the halogen increases the negative inductive effect of the halogen decreases. hence resulting in an increase in the bond length value of halogen as the size increases [13]. The trend is as follows C6–F18 < C6–Cl17 < C6–Br16. It is obvious from the bond length data that; the aromatic ring is slightly distorted from the hexagonal structure. These could be due to the substitution effects of the halogen and the methyl group at the para position. The values of bond angles for PX are C6–C1–C2, C5–C4–C3 (117.6) are reduced than that of a benzene ring but the bond values C1–C6–C5, C4–C3–C2, C1–C2–C3, C6–C5–C4 (121.2) are enlarged. For DFPX, C6–C1–C2, C5–C4–C3 (116.1) are reduced than that of a benzene ring but the bond values C6–C5–C4, C1–C2–C3 (120.3), C1–C6–C5, C4–C3–C2 (123.6) are enlarged. For 2,5 DCPX C6–C1–C2, C5–C4–C3 (116.4) are reduced than that of a benzene ring but the bond values C6–C5–C4, C1–C2–C3 (121.4), C1–C6–C5, C4–C3–C2 (122.2) are enlarged. For 2,5 DBPX C6–C1–C2, C5–C4–C3 (116.3) are reduced than that of a benzene ring but the bond values C6–C5–C4, C1–C2–C3 (121.5), C1–C6–C5, C4–C3–C2 (122.2) are enlarged [14]. Therefore, it is observed that the halogen substitution on p-xylene increase the bond angles but the effect is reduced as the size of the halogen increases. It is also observed from the dihedral angles that all the compounds studied are supported in the planar structure of the aromatic ring.

**Table 1:** Optimized Geometrical Parameters of the Studied Compounds (Bond Angles) Calculated by B3LYP Method with 6-311+G (d, p) basis set with VEDA 4.

Para-Xylene		3,6-Difluoro-Para-xylene		3,6-Dichloro-Para-xylene		3,6-Dibromo-Para-xylene	
Bond Angle	Value	Bond Angle	Value	Bond Angle	Value	Bond Angle	Value
C6–C1–C2	117.6	C6–C1–C2	116.1	C6–C1–C2	116.4	C6–C1–C2	116.3
C6–C1–C11	58.8	C6–C1–C9	57.8	C6–C1–C9	57.7	C6–C1–C9	57.6
C2–C1–C11	58.8	C2–C1–C9	58.3	C2–C1–C9	58.7	C2–C1–C9	58.7
C1–C6–C5	121.2	C1–C6–C5	123.6	C1–C6–C5	122.2	C1–C6–C5	122.2
C1–C6–H10	119.4	C1–C6–F18	118.2	C1–C6–Cl17	119.7	C1–C6–Br18	120.1
C5–C6–H10	119.5	C5–C6–F18	118.1	C5–C6–Cl17	118.0	C5–C6–Br18	117.7
C6–C5–C4	121.2	C6–C5–C4	120.3	C6–C5–C4	121.4	C6–C5–C4	121.5
C6–C5–H9	119.3	C6–C5–H8	119.1	C6–C5–H8	119.2	C6–C5–C4	119.4
C5–C4–C3	117.6	C5–C4–C3	116.1	C5–C4–C3	116.4	C5–C4–C3	116.3
C5–C4–C15	58.8	C5–C4–C13	58.3	C5–C4–C13	58.7	C5–C4–C13	58.7
C3–C4–C15	58.8	C3–C4–C13	57.8	C3–C4–C13	57.7	C3–C4–C13	57.6
C4–C3–C2	121.2	C4–C3–C2	123.6	C4–C3–C2	122.2	C4–C3–C2	122.2
C4–C3–H8	119.4	C4–C3–F17	118.2	C4–C3–Cl18	119.7	C4–C3–Br17	120.1
C2–C3–H8	119.3	C2–C3–F17	118.1	C2–C3–Cl18	118.1	C2–C3–Br17	117.7
C1–C2–C3	121.2	C1–C2–C3	120.3	C1–C2–C3	121.4	C1–C2–C3	121.5
C1–C2–H7	119.4	C1–C2–H7	120.6	C1–C2–H7	119.4	C1–C9–H7	117.1
C1–C11–H16	9.1	C1–C9–H15	9.4	C1–C9–H15	9.2	C1–C9–H15	9.1
C1–C11–H17	9.5	C1–C9–H14	9.4	C1–C9–H14	9.2	C1–C9–H14	9.1
C1–C11–H18	9.1	C1–C9–H16	8.9	C1–C9–H16	9.4	C1–C9–H16	9.5
H16–C11–H17	15.10	H15–C9–H14	15.9	H15–C9–H14	15.9	H15–C9–H14	15.9
H16–C11–H18	16.02	H15–C9–H16	16.0	H15–C9–H16	16.0	H15–C9–H16	16.0
H17–C11–H18	15.9	H14–C9–H16	16.0	H14–C9–H16	16.0	H14–C9–H16	16.0
C4–C15–H12	9.5	C4–C13–H11	9.4	C4–C13–H11	9.2	C4–C13–H11	9.1
C4–H15–H13	9.1	C4–C13–H10	9.4	C4–C13–H10	9.2	C4–C13–H10	9.1
C4–H15–H14	9.1	C4–C13–H12	8.9	C4–C13–H12	9.4	C4–C13–H12	9.5
H12–C15–H13	15.9	H11–C13–H10	15.9	H11–C13–H10	15.9	H11–C13–H10	15.9
H12–C15–H14	15.9	H11–C13–H12	16.1	H11–C13–H10	16.0	H11–C13–H12	16.1
H13–C15–H14	16.1	H10–C13–H12	16.1	H10–C13–H12	16.0	H10–C13–H12	16.1

**Table 2:** Optimized Geometrical Parameters of the Studied Compounds (Bond Length) Calculated by B3LYP Method with 6-311+G (d, p) basis set and VEDA 04.

Para- Xylene		3,6-Difluoro-Para-xylene		3,6-Dichloro-Para-xylene		3,6-Dibromo-Para-xylene	
Bond Length	Value	Bond Length	Value	Bond Length	Value	Bond Length	Value
C1–C6	1.398	C1–C6	1.392	C1–C6	1.398	C1–C6	1.399
C1–C2	1.398	C1–C2	1.398	C1–C2	1.398	C1–C2	1.399
C1–C11	4.351	C1–C9	4.366	C1–C9	4.368	C1–C9	4.371
C6–H10	1.086	C6–F18	1.361	C6–Cl17	1.763	C6–Br18	1.923
C5–C4	1.398	C5–C4	1.398	C5–C4	1.398	C5–C4	1.399
C5–H9	1.086	C5–H8	1.084	C5–H8	1.083	C5–H8	1.083
C4–C3	1.398	C4–C3	1.392	C4–C3	1.398	C4–C3	1.397
C4–C15	4.351	C4–C13	4.366	C4–C13	4.368	C4–C13	4.371
C3–C2	1.393	C3–C2	1.385	C3–C2	1.39	C3–C2	1.39
C3–H8	1.086	C3–F17	1.361	C3–Cl18	1.763	C3–Br17	1.923
C2–H7	1.086	C2–H7	1.084	C2–H7	1.083	C2–H7	1.083
C11–H16	6.347	C9–H15	6.345	C9–H15	6.355	C9–H15	6.36
C11–H17	6.328	C9–H14	6.345	C9–H14	6.355	C9–H14	6.36
C11–H18	6.347	C9–H16	6.35	C9–H16	6.336	C9–H16	6.334
C15–H12	6.328	C13–H11	6.345	C13–H11	6.355	C13–H11	6.36
C15–H13	6.347	C13–H10	6.345	C13–H10	6.355	C13–H10	6.36
C15–H14	6.347	C13–H12	6.35	C13–H12	6.336	C13–H12	6.334

**Table 3:** Optimized Geometrical Parameters of the Studied Compounds (Dihedral Angle) Calculated by B3LYP Method with 6-311+G (d, p) basis set and VEDA 04.

Para-Xylene		3,6-Difluoro-Para-xylene		3,6-Dichloro-Para-xylene		3,6-Dibromo-Para-xylene	
Dihedral Angle	Value	Dihedral Angle	Value	Dihedral Angle	Value	Dihedral Angle	Value
C11–C1–C6–H10	-18059	C2–C1–C6–C5	-0.001	C2–C1–C6–C5	0	C2–C1–C6–C5	-0.001
C6–C1–C2–C3	0.213	C2–C1–C6–F18	-179.996	C2–C1–C6–Cl17	-180.005	C2–C1–C6–Br18	-180.001
C6–C1–C2–H7	-179.9	C9–C1–C6–C5	0	C9–C1–C6–C5	0.001	C9–C1–C6–C5	-0.001
C11–C1–C2–C3	0.627	C9–C1–C6–F18	-179.996	C9–C1–C6–Cl17	-180.004	C9–C1–C6–Br18	-180.001
C11–C1–C2–H7	-179.461	C6–C1–C2–C3	0.001	C6–C1–C2–C3	0	C6–C1–C2–C3	0.001
C6–C1–C11–H16	-28.433	C6–C1–C2–H7	-179.998	C6–C1–C2–H7	-180.001	C6–C1–C2–H7	-179.999
C6–C1–C11–H17	89.786	C9–C1–C2–C3	0	C9–C1–C2–C3	-0.001	C9–C1–C2–C3	0.001
C6–C1–C11–H18	-151.946	C9–C1–C2–H7	-179.999	C9–C1–C2–H7	-180.002	C9–C1–C2–H7	-179.999
C2–C1–C11–H16	-208.054	C6–C1–C9–H15	58.219	C6–C1–C9–H15	60.262	C6–C1–C9–H15	60.938
C2–C1–C11–H17	-89.78	C6–C1–C9–H14	-58.215	C6–C1–C9–H14	-60.262	C6–C1–C9–H14	-60.803
C2–C1–C11–H18	28.483	C6–C1–C9–H16	-179.998	C6–C1–C9–H16	-179.993	C6–C1–C9–H16	-179.939
C1–C6–C5–C4	0,220	C2–C1–C9–H14	-238.215	C2–C1–C9–H14	-240.264	C2–C1–C9–H14	-240.804
C1–C6–C5–H9	-179.868	C2–C1–C9–H16	-121.782	C2–C1–C9–H16	-119.732	C2–C1–C9–H16	-119.063
H10–C6–C5–C4	-179.168	C1–C6–C5–C4	0.001	C1–C6–C5–C4	0	C1–C6–C5–C4	0.001
H10–C6–C5–H9	0.045	C1–C6–C5–H8	-179.998	C1–C6–C5–H8	-180.001	C1–C6–C5–H8	-179.998
C6–C5–C4–C3	-0.213	F18–C6–C5–C4	-180.004	Cl17–C6–C5–C4	-179.995	Br18–C6–C5–C4	-179.999
C6–C5–C4–C15	-0.627	F18–C6–C5–H8	-0.003	Cl17–C6–C5–H8	0.004	Br18–C6–C5–H8	0.001
H9–C5–C4–C3	-180.125	C6–C5–C4–C3	-0.001	C6–C5–C4–C3	0	C6–C5–C4–C3	-0.001
H9–C5–C4–C15	-180.539	C6–C5–C4–C13	0	C6–C5–C4–C13	0.001	C6–C5–C4–C13	-0.001
C5–C4–C3–C2	0.213	H8–C5–C4–C3	-180.002	H8–C5–C4–C3	-179.999	H8–C5–C4–C3	-180.001
C5–C4–C3–H8	-179.875	H8–C5–C4–C13	-180.001	H8–C5–C4–C13	-179.998	H8–C5–C4–C13	-180.001
C15–C4–C3–C2	0.627	C5–C4–C3–C2	0.001	C5–C4–C3–C2	0	C5–C4–C3–C2	0.001
C15–C4–C3–H8	-179.461	C5–C4–C3–F17	-180.004	C5–C4–C3–Cl18	-179.995	C5–C4–C3–Br17	-179.999
C15–C4–C3–H12	-212.981	C13–C4–C3–C2	0	C13–C4–C3–C2	-0.001	C13–C4–C3–C2	0.001
C5–C4–C15–H13	-151.946	C13–C4–C3–F17	-180.005	C13–C4–C3–Cl18	-0.001	C13–C4–C3–Br17	-179.999
C5–C4–C15–H14	-28.483	C13–C4–C3–H10	-204.907	C13–C4–C3–H10	-205.053	C13–C4–C3–H10	-205.154
C3–C4–C15–H12	-89.786	C5–C4–C13–H11	-121.785	C5–C4–C13–H11	-119.736	C5–C4–C3–H11	-119.196
C3–C4–C15–H13	28.483	C5–C4–C13–H12	-0.002	C5–C4–C13–H12	-0.006	C5–C4–C13–H12	-0.001
C3–C4–C15–H14	-208.054	C3–C4–C13–H10	-58.219	C3–C4–C13–H10	-60.262	C3–C4–C13–H10	-60.938
C4–C3–C2–C1	-0.22	C3–C4–C13–H11	58.215	C3–C4–C13–H11	60.262	C3–C4–C13–H11	-60.803
C4–C3–C2–H7	-180.132	C4–C3–C2–C1	-0.001	C4–C3–C2–C1	0	C4–C3–C2–C1	-0.001
H8–C3–C2–C1	-180.132	C4–C3–C2–H7	-180.002	C4–C3–C2–H7	-179.999	C4–C3–C2–H7	-180.002
H8–C3–C2–H7	-0.045	F17–C3–C2–C1	-179.996	Cl18–C3–C2–C1	-180.005	Br17–C3–C2–C1	-180.001
C2–C1–C6–C5	-0.213	F17–C3–C2–H7	0.0003	Cl18–C3–C2–H7	-0.004	Br17–C3–C2–H7	-0.001
C2–C1–C6–H10	-180.125	C3–C4–C13–H12	-180.002	C3–C4–C13–H12	-180.002	C3–C4–C13–H12	-180.061
C11–C1–C6–C5	-0.627	C2–C1–C9–H15	-121.782	C2–C1–C9–H15	-119.739	C2–C1–C9–H15	-119.603

### 3.2 Vibrational analysis

The goal of the vibrational analysis is to determine the vibrational modes associated with relevant and specific molecular structures of the calculated compounds studied. The maximum number of potentially active observable fundamentals of a non-linear molecule which contains N atoms is equal to (3N-6) normal modes of vibration [15]. Hence, the PX molecule has 18 atoms with 48 (17 Stretch Vibrations, 16 bend Vibrations, 11 torsional Vibrations, 4 Out of Plane vibrations) normal modes of vibration. DFPX, also, have 18 atoms with 48 normal modes of vibration (17stretch vibrations, 16 bend vibrations, 11 torsional vibrations, 4 out-of-plane vibrations). DCPX has 18 atoms with 48 (17 stretch vibrations, 16 bend vibrations, 9 torsional vibrations, 6 out-of-plane vibrations) normal modes of vibration. DBPX has 18 atoms and so undergoes 48 modes of vibration similar to that of DCPX except that chlorine is replaced with bromine. This is represented in Tables 4, 5, 6, and 7, and it could be seen that, not all vibrations are active both in Raman and Infrared absorption. The calculated frequencies using the B3LYP method with 6-311+G basis set along with their IR and Raman intensities, probable assignments and potential energy distribution (PED) are summarized in Tables 4, 5, 6, 7 and their corresponding spectra in Figure S1 to S4 of supporting information.

**Table 4:** Vibrational Assignments of Calculated Frequencies of PX Calculated by B3LYP Method with 6-311+G (d, p) basis set.

Para-Xylene			
Frequency	IR Intensity	Raman activity	Assignment of ped (%)
3166	0	0	vCH(82)+asyvCH(10)
3162	46.75	0	vCH(81)+vCH(10)
3146	0	129.06	vCH(100)
3146	24.26	0	asyvCH(10)+asyvCH(81)
3097	0	124.98	vCH(75)
3097	35	0	vCH(75)
3071	40.87	0	vCH(84)
3071	0	174.82	vCH(84)
3018	0	504.61	vCH(87)
3018	69.48	0	asyvCH(87)
1656	0	37.71	asyvCC(63)+asybHCC(20)+asybCCC(12)
1613	0	5.09	vCC(71)
1547	29.69	0	bHCC(58)+asybCCC(11)
1501	19.49	0	bHCH(72)+asytHCCC(21)
1490	14.14	0	bHCH(72)+asytHCCC(21)
1489	0	20.78	asybHCH(74)+asytHCCC(24)
1488	0	14.21	bHCH(72)+asytHCCC(21)
1435	0	0	vCC(35)+bHCC(18)+bCCC(14),asybCCC(10)
1415	0	32.9	bHCH(94)
1411	1.25	0	bHCH(91)
1341	0	2.69	bHCC(52)+bHCC(19)
1323	0.1	0	vCC(79)
1237	3.19	0	vCC(30)+bHCC(34)+bCCC(22)
1222	0	32.11	asyvCC(91)
1208	0	6.74	asyvCC(14)+bHCC(72)
1140	7.44	0	vCC(29)+bHCC(10)+asybHCC(40)
1063	17.97	0	asybHCH(21)+tHCCC(63)
1061	0	3.94	bHCH(18)+tHCC(60)+tCCCC(11)+OUTCCCC(11)
1038	1.4	0	bCCC(81)
1024	0	1.09	bHCH(19)+asytHCCC(65)
988	0	0	vCC(13)+asybHCH(19)+tHCCC(52)
978	0	0	asytHCCC(83)+tCCCC(46)
955	0	0.28	asytHCCC(73)+tCCCC(11)+OUTCCCC(11)
848	0	0.75	tHCCC(100)
836	0	38.4	vCC(74),asybCCC(15)
811	42.49	0	asytHCCCC(87)
728	0.41	0	asyvCC(52)+bCCC(35)
7222	0	0.25	tHCCC(12)+tCCCC(69)+OUTCCCC(69)
659	0	5.88	vCC(11),bCCC(79)
496	21.14	0	asyOUTCCCC(92),asytCCCC(92)
464	0	9.87	asyvCC(15)+vCC(17)+bCCC(67)
416	0.02	0	tHCCC(16)+tCCCC(84)
387	0	0.16	bCCC(12)+bCCC(81)
308	0	2.19	asyOUTCCCC(85)+asybCCC(85)
286	0.7	0	bCCC(82)
135	2.18	0	asyOUTCCCC(88)+asytCCCC(88)
56	0	1.63	tHCCC(100)
43	0.53	0	tHCCC(97)

**Table 5:** Vibrational Assignments of Calculated Frequencies of DFPX Calculated by B3LYP Method with 6-311+G (d, p) basis set.

DFPX			
Frequency	IR Intensity	Raman Activity	Assignment of PED (%)
3191	0	198	vCH(100)
3189	4.08	0	asyvCH(100)
3114	0	126.37	asyvCH(21)+vCh(79)
3114	28.1	0	asyvCH(21)+vCh(79)
3084	23.23	0	asyvCH(100)
3084	0	182.81	vCH(100)
3034	0	512.4	vCH(79)+vCH(21)
3034	46.67	0	asyvCH(79)+asyvCH(21)
1672	0	47.43	asyVCC(75)
1621	0	4.15	asyvCC(69)+asybCCC(11)+asybCCF(11)
1534	168.68	0	vCC(43)+vFC(43)+vCC(43)+bHCC(32)
1505	21.97	0	bCCC(10)+bHCH(44)+bHCH(17)+asytHCCC(12)
1487	0	17.92	bHCH(55)+asytHCCC(15)
1481	15.65	0	bHCH(70)+tHCCC(17)
1481	0	16	bHCH(70)+asytHCCC(19)
1430	25.24	0	asyvCC(12)+asyvFC(12)+bCCC(29)+asybHCH(23)
1419	0	28.82	bHCH(82)+bHCH(11)
1412	19.04	0	asybCCC(21)+bHCH(30)
1330	2.45	0	vCC(80)
1317	0	35.64	vCC(89)+vFC(89)
1255	0	1.74	bHCC(74)
1209	84.54	0	asyvCC(32)+asyvFC(32)+asybCCC(26)
1178	101.46	0	asyvCC(24)+asyvFC(24)+asyvCC(24)+bHCC(52)
1092	0	2.41	asyvCC(70)+asyvFC(70)
1064	3.73	0	asybHCH(24)+asytHCCC(55)
1056	0	0.02	asytHCCC(63)+bHCH(23)
1031	0	1.43	asyvCC(11)+asybHCH(13)+tHCCC(35)
1009	32.1	0	bHCh(16)+tHCCC(36)
895	37.88	0	asytHCCC(76)+asyOUTFCCC(10)+asyOUTCCCC(10)
867	0	0.05	tHCCC(79)+tCCCC(11)+OUTCCCC(11)+tCCCC(11)
831	40.26	0	vCC(75)+vFC(75)
754	0	27.16	vCC(61)+asybCCC(31)+asybCCF(31)
708	0	0.43	asytHCCC(13)+tCCCC(74)+OUTCCCC(74)+tCCCC(74)+OUTFCCC(74)
680	24.78	0	asyvCC(51)+asyvFC(51)+bCCC(31)
639	0.73	0	OUTFCCC(73)+OUTCCCC(73)
585	0	3.93	asybCCC(77)+asybCCF(77)
498	0	14.05	vCC(34)+bCCC(47)+bCCF(47)
464	6.38	0	tCCCC(84)+OUTCCCC(84)
432	0	3.17	vCC(12)+vFC(12)+bCCC(68)+bCCC(13)+bCCF(13)
388	0	2.05	OUTCCCC(87)+OUTFCCC(87)
338	5.6	0	asybCCC(13)+bCCF(75)
269	3.16	0	bCCC(78)
265	0	0.73	asybCCC(94)+asybCCF(94)+asybCCC(94)+asybCCF(94)
260	0	2.02	OUTCCCC(78)+tCCCC(78)+OUTFCCC(78)
178	0	0	tCCCC(77)+OUTFCCC(77)+tCCCC(77)+OUTCCCC(77)
119	3.56	0	tCCCC(85)
83	0	0.91	tHCCC(10)+tHCCC(79)
82	0.32	0	tHCCC(80)

**Table 6:** Vibrational Assignments of Calculated Frequencies of DCPX Calculated by B3LYP Method with 6-311+G (d, p) basis set.

DCPX			
Frequency	IR Intensity	Raman Activity	Assignment of PED (%)
3191	0	165.4	vCH(99)
3189	3.74	0	vCH(100)
3115	29.79	0	asyvCH(20)+vCH(79)
3115	0	116.49	asyvCH(20)+vCH(20)
3084	19.74	0	vCH(100)
3084	0	156.88	vCH(100)
3033	0	462.8	vCH(80)+vCH(20)
3033	36.68	0	vCH(79)+vCH(20)
1638	0	38.64	asyvCC(74)+asyb(12)
1583	0	18.84	asyvCC(66)
1509	78.96	0	bCCC(26)+asybCCC(39)
1499	26.08	0	asybHCH(53)+tHCCC(23)
1484	0	8.1	asybHCH(57)+asytHCCC(22)
1483	17.62	0	bHCH(68)+tHCCC(19)
1482	0	16.69	bHCH(69)+asytHCCC(9)
1421	2.17	0	bHCH(77)
1420	0	28.5	bHCH(81)
1382	21.1	0	vCC(65)
1306	3.37	0	vCH(77)
1284	0	0.05	bHCC(79)
1246	0	34.31	asyvCC(90)
1211	2.36	0	vCC(22)+bHCC(12)+bHCC(41)
1084	124.97	0	vClC(11)+bCCC(12)+bHCCC(11)+bCCC(56)
1064	5.19	0	asybHCH(24)+asytHCCC(62)
1057	0	0.03	bHCH(24)+asytHCCC(65)
1042	0	0.75	bHCH(15)+tHCCC(65)
1007	30.23	0	asybHCH(14)+tHCCC(54)
942	0	7.53	vCC(80)+vClC(80)+bCCC(11)
892	23.04	0	asytHCCC(79)
878	0	0.02	tHCC(83)
770	26.66	0	vCC(51)+asyvClC(12)+asyvCCC(25)
718	0	18.88	vCC(15)+asyvClC(26)+bCCC(67)+bCCC(19)+bCCCl(19)
703	0	0.48	asytHCCC(11)+asyOUTHCCCC(11)+OUTCCCC(81)+tCCCC(81)+OUTClCCC(81)
607	0	0	asytCCCC(74)+OUTClCCC(74)
531	25.66	0	vClC(67)+asybCCC(19)
524	0	4.92	asybCCC(79)+asybCCC(79)
472	0	11.53	vClC(17)+vCC(17)+vCC(10)+vClC(10)+bCCC(30)+bClCC(30)
454	6.56	0	asytHCCC(12)+asytCCCC(12)+asytClCCC(15)+OUTClCCC(15)+asytCCCC(67)+OUTCCCC(67)
344	0	0.36	OUTCCCC(89)+OUTClCCC(89)
321	0	10.21	vClC(51)+vCC(51)+bCCC(38)
288	3.69	0	bCCC(76)
240	0	1.63	bCCC(89)+bCCCl(89)
239	0	1.62	OUTCCCC(81)+tCCCC(81)
221	0.89	0	bCCCl(86)
161	0.39	0	tHCCC(55)
145	0	0.93	asytHCCC(89)
135	1.34	0	asytHCCC(41)+asyOUTCCCC(49)+asyOUTClCCC(49)
85	1.14	0	tCCCl(13)+OUTClCCC(13)+OUTCCCC(13)+asytCCCC(70)+asyOUTClCCC(70)+tCCCC(15)+OUTCCCC(15)

**Table 7:** Vibrational Assignments of Calculated Frequencies of DBPX Calculated by B3LYP Method with 6-311+G (d, p) basis set.

DBPX			
Frequency	IR Intensity	Raman Activity	Assignment of PED (%)
3192	0	149.5	vCh(99)
3190	2.99	0	vCh(99)
3113	31.37	0	asyvCH(21)+vCH(79)
3113	0	116.35	asyvCH(21)+vCH(79)
3085	18.08	0	vCH(100)
3085	0	142.53	vCH(100)
3033	0	441.17	vCH(79)+vCH(21)
3033	33.35	0	vCH(79)+vCH(21)
1628	0	36.33	asyvCC(79)+asybHCC(10)
1570	0	21.01	asyvCC(68)+bHCH(13)
1502	65.24	0	vCC(14)+bHCC(52)+bHCH(52)
1496	30.78	0	vCC(11)+asybHCC(57)+asybHCH(57)+asybCCC(12)
1482	0	6.87	asybHCH(64)+asytHCCC(20)
1481	20.27	0	bHCH(75)+tHCCC(24)
1481	0	16.54	asybHCH(79)+tHCCC(17)
1420	3.03	0	bHCH(93)
1420	0	26.44	bHCH(95)
1371	17.54	0	vCC(16)+bCCC(30)
1299	4.41	0	vCC(81)
1285	0	1.04	vCC(11)+asybHCC(76)
1238	0	36.2	vCC(92)
1212	3.89	0	vCC(51)+asybHCC(18)+asybHCH(18)
1065	121.73	0	asyvCC(14)+bCCC(54)
1063	4.25	0	asybHCH(20)+tHCCC(61)
1055	0	0.36	bHCH(21)+asytHCCC(52)
1041	0	1.69	bHCH(16)+tHCCC(59)
1003	32.9	0	asybHCC(12)+asybHCH(12)+asybHCC(11)+asybHCH(11)+asytHCCC(30)
908	0	9.06	vCC(51)+asyvBrC(23)+asybCCC(14)
886	20.03	0	asytHCCC(77)+asyOUTCCCC(11)+asytCCCC(11)+asyOUTBrCCC(11)
872	0	0.18	tHCCC(86)
758	25.7	0	vCC(51)+asybCCC(29)
702	0	17.57	vCC(11)+vBrC(11)+bCCC(56)
682	0	0.24	asyOUTCCCC(50)+asytCCCC(50)+asyOUTBrCCC(50)+OUTCCCC(10)+tCCCC(10)+OUTBrCCC(10)+OUTCCCC(15)+tCCCC(15)
584	0.08	0	OUTCCCC(74)+OUTBrCCC(74)
503	0	5.48	bCCC(82)+bCCBr(82)+bCCC(82)
467	0	9.19	vCC(25)+bCCC(57)
446	6.58	0	asytHCCC(13)+OUTCCCC(26)+tCCCC(26)+OUTBrCCCC(26)+asyOUTCCCC(12)+asytCCCC(12)+asyOUTBrCCC(12)+OUTCCCC(46)+tCCCC(46)
436	9.87	0	vBrC(66)+bCCC(11)+asybCCC(85)
331	0	0.8	OUTCCCC(85)+OUTBrCCC(85)
270	4.3	0	vCBr(17)+bCCC(64)
221	0	1.6	asyOUTCCCCC(69)+asytCCCC(69)+asyOUTBrCCC(69)
211	0	7.71	vBrC(57)+asybCCC(14)+asybCCC(12)
208	0	1.13	bCCC(15)+bCCC(75)+bCCBr(75)+bCCC(75)
163	0.24	0	bCCBr(90)
154	0.68	0	tHCCC(44)+asyOUTCCCC(38)+asytCCCC(38)+asyOUTBrCCC(38)
138	0	1.1	asytHCCC(12)+asytHCCC(58)+OUTCCCC(13)+tCCCC(13)+OUTBrCCC(13)
131	1.65	0	asytHCCC(35)+asyOUTCCCC(31)asytCCCC(31)+asyOUTBrCCC(31)
64	0.44	0	asytCCCC(90)+asyOUTBrCCC(90)

#### 3.2.1 C–H vibrations

The PX molecule is a di-substituted aromatic structure. DFPX, DCPX, and DBPX are all tetra-substituted molecules. PX causes 3 C–H stretching vibrations. DFPX causes 2 C–H stretching vibrations. DCPX causes 2 C–H stretching vibrations. The characteristic region for the ready identification of the C–H stretching vibrations for aromatic rings is in the range 3300–3000cm^−1^ [16]. PX stretching C–H vibrations are calculated to be 3146, 3162, 3166cm^−1^ which corresponds to other theoretical values from literature [17]. DFPX stretching vibrations are also calculated to be 3189, 3191cm^−1^. DCPX stretching vibrations are calculated to be the same as that of DFPX i.e. 3189, 3191cm^−1^ for DCPX. Finally, DBPX C–H stretching vibrations are also calculated to be 3192 and 3190cm^−1^. It is observed from the PED analysis that all the vibrational modes mentioned are pure C–H stretching because of the PED percent which is greater than 99%.

#### 3.2.2 C–C vibrations

The ring C–C and ring C=C stretching vibrations (semi-circle stretching region) generally appear in the region 1625-1400cm/1 and 1380-1280cm^−1^ [18]. The PX ring C–C vibrations contain frequencies that occur in the range (464–1435) cm^−1^. The vibrations occurring in the region other than that specified for ring C–C and C=C vibrations are assigned to C–C in-plane vibrations and C–C out of plane vibrations. DFPX C–C vibrations contain frequencies that occur in the range (432–1673) cm^−1^. DCPX C–C vibrations contain frequencies that occur in the range (472–1638). The values of frequencies obtained for ring C–C and C=C vibrations are almost equal when compared to the work by Venkatesh *et. al.* [1]. DBPX C–C vibrations contain frequencies that occur in the range (466–1628) cm/1.

#### 3.2.3 C-X vibrations (X = F, Cl, Br)

Fluorine substituted aromatic compounds give stretching bands in the region 1270-1100 cm^−1^ [19, 20]. The C–Cl stretching is generally observed in the region 800cm^−1^ -500cm^−1^ which depends on the configuration and conformation of the compound. DCPX C–Cl stretching calculated vibrations are (718,472,327,1084,531)cm^−1^. From the vibrational frequencies of calculated C–Cl stretch vibrations, the C–Cl out-of-plane vibrations appear at 531,472,327cm^−1^. DFPX C–F stretching calculated vibrations are (1317, 1030, 831, 552) cm^−1^. C–F in-plane bending vibration is expected in the range (420-254) cm^−1^. The C–F out-of-plane bending vibrations are observed in the range (520-107) cm^−1^. The out-of-plane vibrations assigned at 432 cm^−1^ by the B3LYP/6-311+G method agree with the recorded data [21, 22]. DBPX C–Br stretching calculated vibrations are (436,270,908,702 and 211) cm^−1^.

#### 3.2.4 Methyl group vibrations

In PX, DFPX, DCPX, and DBPX they are groups substituted in the first and fourth position of the aromatic ring. The asymmetric C–H stretching mode is expected around 2980 and symmetric stretching is expected at 2870 [23]. PX has six stretching vibrations and C–H stretching vibrations for the group include (3018,3071,3097). DFPX has six stretching vibrations and C–H stretching vibrations for the group include (3084,3114). DCPX has six stretching vibrations and C–H stretching vibrations for the group include (3084,3115). DBPX has six symmetric stretching vibrations and C–H stretching vibrations for the group include (3085,3113). The theoretically calculated values approximately correspond to the values found in literature [17].

With the VEDA Software, it is possible to determine the maximum intensity, frequency value for the maximum intensity and its corresponding mode of vibration. Thus, the maximum infrared intensity for Para xylene observed is 69.48 and its frequency value is 3018 and it is due to asymmetric stretching while the maximum infrared intensity for 3,6-DFPX is 168.68 and the frequency value is 1534 which is due to two normal modes of vibration, being symmetrical C–C stretching and H–C–C bending. The maximum infrared intensity for 3,6-DCPX is 124.97 and the frequency value is 1086 and is due to 4 normal modes of vibration. (a) symmetrical Cl–C stretch (b) bend C–C–C (c) asymmetric bend HCC (d) bend C–C–C. The maximum infrared intensity for 3,6 DBPX is 121.73 and the frequency value is 1064 which is due to two normal modes of vibration. (a) asymmetrical C–C stretching and (b) bend C–C–C (see Figures 1, 2, 3, and 4).

**Figure 1:** Optimized structure and the orbitals involved in the electronic transition of PX, for the Highest Occupied Molecular Orbital (HOMO) and Lowest Unoccupied Molecular Orbital (LUMO) respectively.

**Figure 2:** Optimized structure and the orbitals involved in the electronic transition of DFPX, for the Highest Occupied Molecular Orbital (HOMO) and Lowest Unoccupied Molecular Orbital (LUMO) respectively.

**Figure 3:** Optimized structure and the orbitals involved in the electronic transition of DCPX, for the Highest Occupied Molecular Orbital (HOMO) and Lowest Unoccupied Molecular Orbital (LUMO) respectively.

**Figure 4:** Optimized structure and the orbitals involved in the electronic transition of DBPX, for the Highest Occupied Molecular Orbital (HOMO) and Lowest Unoccupied Molecular Orbital (LUMO) respectively.

### 3.3 UV-vis spectroscopic analysis

The electronic activities of PX, DBPX, DCPX and DFPX have been estimated by TD-DFT/B3LYP/6-311+G(d,p). The wavelengths (λ), oscillator strengths (f) and energies for excitation (E) are listed in Table 8 and the theoretical ultraviolet spectrum of these compounds is shown in Figure 5. The TD-DFT calculation revealed three different transitions for each of the studied molecules. As shown in Figure 5, the major transitions are: PX 5.7194ev with λmax of 216.78nm and an oscillator strength (f) of 0.0550 while DBPX has its major transitions at 4,8679ev with a corresponding λmax of 254.70nm and an oscillator strength of 0.0227. the major transition corresponding to DCPX was observed at 5.4786ev with λmax of 226.37nm and oscillator strength of 0.1075 while that for DFPX was seen at 5.0903ev with λmax of 243.57nm and an oscillator strength of 0.0430. As a result of the negligible or zero oscillator strengths of other excitations, their transitions or excitations do not have detectable contributions to the UV-Vis spectrum and as such are not included. It can be inferred from the result that the theoretical excitation wavelength of the studied compounds is in the order DBPX > DFPX > DCPX > PX, it can also be seen that DBPX had the lowest vertical excitation energy while P-xylene had the highest excitation energy. The order of theoretical oscillator strength as observed from the result is 0.055 for PX > 0.0430 for DFPX >0.0227 for DBPX which is in turn greater than 0.1075 for DCPX. These transitions correspond to π-π∗ transitions respectively. The UV spectra was plotted with the help of mutiwfn and their major contributions were as well calculated with the help of multiwfn program [11]. The interactions that exits in molecules between electron donors and acceptors is often in concomitant with the formation of an intensely coloured charge transfer complex that mostly absorbs radiation in the UV-vis region [24]. The formation of charge transfer complex in compounds is caused by the presence of delocalized electrons in compounds and this is seen to improve the biological activities of most compounds [19]. It can be observed from the results that the electronic transition between the HOMO and LUMO energy levels is predominantly found within the UV region of the spectrum which is an indication that the studied compounds will be inactive in the visible region and also that these compounds in their pure state are expected to colorless.

**Table 8:** Calculated wavelengths of absorption, % contribution from each transition, transition energies, and oscillator strength computed at the B3LYP/6-311G+(d,p) level.

P-Xylene				
λ(nm)	E(eV)	F	Major contributions	Assignment
216.78	5.7194	0.0550	H-L67.74 %	π → π∗
241.67	5.1303	0.0050	H-L70.33%	
DBPX				
254.70	4.8679	0.0227	H-L40.68%	π → π∗
236.28	5.2474	0.0013	H-L94.67%	
DCPX				
251.64	4.9271	0.0179	50.23%	π → π∗
226.31	5.4786	0.1075	44.56%	
DFPX				
243.57	5.0903	0.0430	54.70%	π → π∗
211.37	5.8657	0.0259	54.70%

**Figure 5:** Simulated UV-Vis spectra of 3,6-dichloro, 3,6-dibromo, 3,6-difluoro-P-xylene and P-xylene calculated with B3LYP/6-311+G(d,p) basis sets. The curves correspond to molar absorption coefficient broadened by calculated excitation energies and oscillator strengths.

The frontier molecular orbitals of the compounds are presented in Figure 5 the HOMO of 3,6-difluoro-p-xylene is located over the aromatic ring, the fluorine atom and methyl groups while the LUMO is delocalized over the 4 carbon atoms of the aromatic ring and the carbon atoms of the methyl group substituent. These (HOMO→LUMO ) transitions suggest an electron density transfer from the halogen atom to the C–C bonds of the aromatic ring while the HOMO of P-xylene is delocalized over the aromatic ring and the methyl substituents and the LUMO is located at the C–C double bonds of the aromatic ring; this shows an electron density transfer from the methyl groups to the aromatic ring. The HOMO of 3,6-dichloro-p-xylene is located over the benzene ring, Chlorine atom and methyl groups and the LUMO is delocalized over the ring and the Chlorine atoms indicating strong density around the ring and halogen atoms, the electron density transfer in this case is seen to occur between the carbon atoms of the methyl group and the ring confirming the electron donating properties of the methyl groups and the strong electron withdrawing effect of the Cl atom likewise the HOMO of 3,6-dibromo-p-xylene is located over the ring, halogen atom and the Carbon atom of the methyl group while the LUMO is also located at the ring and Br atom suggesting a strong electron densities in these regions.

### 3.4 NMR analysis

The physical and chemical properties of an atom is often accessed by its paramagnetic shield and this shield is often influenced by the type of atom it's been bonded to directly or indirectly. The physicochemical properties of the two interacting atoms are greatly altered with respect to the electronic densities around the atoms. The asymmetrical displacement of the electron clouds between two bonding atoms and the type of substituent that is bonded to the reacting atoms affects the chemical properties of the developing product [6]. These displacement of electron clouds can be analyzed by observing the chemical shift of the interacting atoms. Generally, the chemical shifts of carbon and hydrogen atoms is dependent on their chemical environment in compounds. The calculated values of the chemical shift of P-xylene, 3,6-dibromo, 3,6-dichloro, and 3,6-difluoro-pxylene have been simulated using B3LYP/6-311+G(d,p) GIAO with TMS as reference and is presented in Table 9 and the corresponding theoretical spectra are presented in Figures S6-S13 of supporting information.

**Table 9:** Calculated ^1^H and ^13^CNMR chemical shift (ppm) of the studied compounds obtained by B3LYP/6-311+G(d,p) GIAO with TMS as reference.

Carbons Atom with position	Chemical shift (ppm) TMS B3LYP/6-311+G(2d,p) GIAO	Hydrogen Atoms with positions	Chemical shift (ppm) TMS B3LYP/6-311+G(2d,p) GIAO
P-Xylene			
1C	140.59	7H	7.23
2C	133. 38	8H	7.23
3C	133. 38	9H	7.23
4C	140.59	10H	7.23
5C	133. 38	12H	2.53
6C	133. 38	13H	2.14
11C	21.64	16H	2.14
15C	21.64	17H	2.14
		18H	2.14
		12H	2.53
DBPX			
1C	142.93	7H	7.4
2C	139	8H	7.4
3C	146.65	10H	2.4
4C	142.93	11H	2.4
5C	139	12H	1.9
6C	146.65	14H	2.4
9C	22.93	15H	2.4
13C	22.93	16H	1.9
DCPX			
1C	141.15	7H	7.23
2C	135.23	8H	7.23
3C	146.4	10H	2. 3
4C	141.15	11H	2. 3
5C	135.23	12H	1.8
6C	146.4	14H	2. 3
9C	21.15	15H	2. 3
13C	21.15	16H	1.8
DFPX			
1C	130	7H	6.9
2C	121	8H	6.9
3C	166.2	10H	2. 35
4C	130	11H	2. 35
5C	121	12H	1.7
6C	166.2	14H	2. 35
9C	16.2	15H	2. 35
13C	16.2	16H	1.7

From literature [25] the experimental chemical shift of aromatic carbon atoms is in the range of 120–190ppm while that of aliphatic chain is constantly behind the aromatic compounds [26] As observed from the results of the studied compounds, the calculated chemical shift of the aromatic ring in P-Xylene is in the range of 133–140ppm and that of DBPX is in the range of 139–140ppm while DCPX had its aromatic chemical shift between 135 -140ppm likewise DFPX had its aromatic chemical shift in the range of 130–166ppm which is in close proximity with the experimental values. The aromatic carbon atoms with halogen atoms directly attached to them had a slightly higher chemical shift than others; the aromatic carbon atom with Br atoms in DBPX had a chemical shift of 146.6ppm while that in DCPX had a chemical shift of 146.4ppm due to the similar electron withdrawing effect of the Br and Cl atoms. The chemical shift of the carbon atoms (C3&C6) of DFPX is seen to be 166.2ppm which is quite higher than others due to the high electronegativity of the fluorine atom. The meta-substitution pattern of the studied compounds can be confirmed from both the ^13^CNMR and ^1^HNMR spectra, the ^13^CNMR spectra gives three peaks in the aromatic region with a degeneracy of 2:2:2 corresponding to two carbon atoms respectively while the proton NMR spectra shows only one peak in the aromatic region with an integration of 2. The aromatic protons in DBPX is seen to have a chemical shift of 7.4ppm while in DCPX it is observed at 7.23ppm and 6.9ppm in DFPX. The methyl group protons 10H,11H,14H and 15H are seen to have a slightly higher chemical shift of 2.4ppm in DBPX, 2.3ppm in DCPX and 2. 35ppm in DFPX than the other two protons (12H and 16H) on the same methyl groups with chemical shifts of 1.9ppm in DBPX, 1.8ppm in DCPX, and 1.7ppm in DFPX as a result of coupling with the halogen substituted carbon atoms. The magnetic equivalence observed in most protons and carbon atoms from the result is due to symmetry in the studied compounds respectively.

### 3.5 Natural bond orbital (NBO) analysis

Natural bond orbital (NBO) analysis affords a proficient technique for studying intra- and intermolecular bonding interactions between bonds and also provides a convenient basis for investigating charge transfer or conjugative interactions in molecules [27]. previous research [28] has reported the electron donor orbitals, electron acceptor orbitals along with their stabilization energy arising from the second-order perturbation theory. The greater the perturbation energy value, the stronger the interaction between the electron donors and the more intense the system is conjugated [29]. The electron density delocalization between the occupied (Lewis) and unoccupied (non-Lewis) NBO orbitals which shows a more stable donor-acceptor interaction can also be obtained from the NBO analysis [24]. The NBO analysis of 3,6-dibromo-p-xylene, 3,6-dichloro-p-xylene, 3,6-difluoro-p-xylene, and p-xylene was conducted using DFT/B3LYp/6-311+G (d, p) basis set with NBO 7.0 program to determine the intramolecular hybridization, conjugative interaction and electron density delocalization of the studied molecules respectively.

The second-order Fock Matrix is conducted to estimate the donor-acceptor interactions in NBO analysis [12]. The second-order perturbation energy values of DBPX, DCPX, DFPX and PX were calculated with respect to the second-order Fock matrix perturbation theory using DFT/B3LYP/6-311+G (d, p) functional. The most interacting NBOs are tabulated in Table 11 corresponding to the studied molecules respectively. Molecular interaction in the studied molecules is observed by a π-π∗, π∗-π∗ transition between C–C orbitals. These interactions are observed as an increase in electron density within the C–C antibonding orbitals of the molecules [30]. the electron densities of the conjugated double and single bond in the ring system are seen to be approximately 1.9e which vividly validates the strong electronic delocalization within the molecules respectively.

Table 10 show the calculated occupancies of natural orbitals (Lewis and non-Lewis type σ and π bonding orbitals). The calculated natural hybrids on atoms are also were given as well. As observed from Table 10, the π(C4–C5) bond is seen to have the lowest occupancy of 1.64757e which is formed from a hybrid $sp^{1.00}$ on carbon 5 and is predominantly contributed by 0.00% s, 99.96% p and 0.04% d character while the σ(C1–C2) bond is formed from a hybrid $sp^{1.95}$ on carbon 2 with 33.88% s, 66.10% p and 0.02% d atomic orbital. The LP(2) Br17 is seen to have an occupancy of 1.97452e and is formed from a hybrid $sp^{99.96}$ on bromine 17 with 0.00% s, 99.99% p, and 0.01% d character. It is apparent from the result that the π(C1–C2) bond has the lowest occupancy of 1.65267 electrons and is formed from a hybrid $sp^{1.00}$ on carbon 2 which is mainly contributed by 0.00% s, 99.95% p and 0.05% d character while the σ(C3–C4) bond with 1.9734e occupancy is formed from a hybrid $sp^{1.55}$ on carbon 4 with 39.18% s, 60.78% p and 0.04% d atomic orbital contribution. The LP(3) Cl17 with 1.93026e occupancy is fashioned from a hybrid $sp^{1.00}$ on chlorine which is a mixture of 0.00% s, 99.97% p and 0.03% d atomic orbital. The πC3-C4 is seen from to have the lowest occupancy of 1.6471e and is made from a hybrid $sp^{1.00}$ on carbon 4 which is principally contributed by 0.00% s, 99.96% p and 0.04% d atomic orbital while the σ(C3–C4) is formed from a hybrid $sp^{1.54}$ on carbon 4 with 39.29% s, 60.68% p and 0.04% d atomic orbital and has an occupancy of 1.97520 electrons. The LP(1) Fl7 is contributed by 70.01% s, 29.98% p, and 0.00% d atomic orbital and is fashioned from a hybrid $sp^{1.43}$ on Fluorine with occupancy of 1.99009 electrons. As observed from Table 10, the π(C1–C6) bond is formed from the $sp^{1.00\;}$ hybrid on carbon 6 which is a combination of 0.00% s, 99.95% p, and 0.04% d atomic orbital. It can also be seen that the π(C2–C3) bond is formed from the hybrid $sp^{1.00}$ on carbon 3 from a combination of 0.00% s, 99.96% p, and 0.04% d atomic orbitals.

**Table 10:** Natural Orbital Occupancies and hybrids of the most interacting NBOs of all the studied compounds calculated by B3LYP method with 6-311+G (d, p) functional.

Donor Lewis-type NOBs	Occupancy	Hybrid	AO(%)
σC1-C2	1.95508	$sp^{1.95}$	s(33.88%)p(66.10%)d(0.02%)
πC1-C6	1.66232	$sp^{1.00}$	s(0.00%)p(99.95%)d(0.05%)
πC3-C4	1.69505	$sp^{1.00}$	s(0.00%)p(99.96%)d(0.04%)
πC4-C5	1.98006	$sp^{1.00}$	s(0.00%)p(99.96%)d(0.04%)
π∗C2–C3	0.38921	$sp^{1.79}$	s(35.74%)p(64.14%)d(0.11%)
LP(3) Br17	1.93740	$sp^{1.00}$	s(0.00%)p(99.98%)d(0.02%)
DCPX			
σC1-C2	1.95874	$sp^{1.93}$	s(34.08%)p(65.88%)d(0.04%)
πC1-C2	1.65267	$sp^{1.00}$	s(0.00%)p(99.95%)d(0.05%)
πC3-C4	1.66032	$sp^{1.00}$	s(0.00%)p(99.98%)d(0.02%)
πC5-C6	1.97755	$sp^{1.82}$	s(35.44%)p(64.52%)d(0.05%)
LP(3)-Cl17	1.93026	$sp^{1.00}$	s(0.00%)p(99.97%)d(0.03%)
LP(3)-Cl18	1.93026	$sp^{1.00}$	s(0.00%)p(99.97%)d(0.03%)
π∗C3–C4	0.41016	$sp^{1.00}$	s(0.00%)p(99.98%)d(0.02%)
π∗C5–C6	0.39388	$sp^{1.00}$	s(0.00%)p(99.95%)d(0.05%)
DFPX			
πC1-C2	1.67649	$sp^{1.00}$	s(0.00%)p(99.94%)d(0.06%)
πC3-C4	1.64731	$sp^{1.00}$	s(0.00%)p(99.96%)d(0.04%)
πC5-C6	1.97846	$sp^{1.90}$	s(34.43%)p(65.52%)d(0.06%)
LP(3)-F17	1.93214	$sp^{1.00}$	s(0.00%)p(99.98%)d(0.02%)
LP(3)-F18	1.93214	$sp^{1.00}$	s(0.00%)p(99.98%)d(0.02%)
PX			
πC1-C6	1.6496	$sp^{1.00}$	s(0.00%)p(99.95%)d(0.04%)
πC2-C3	1.6797	$sp^{1.00}$	s(0.00%)p(99.96%)d(0.04%)
πC4-C5	1.6496	$sp^{1.00}$	s(0.00%)p(99.95%)d(0.04%)
σC11-H12	1.9765	$sp^{3.38}$	s(22.82%)p(77.12%)d(0.06%)
σC15-H17	1.9765	$sp^{1.38}$	s(22.82%)p(77.12%)d(0.06%)
π∗C1–C6	0.3514	$sp^{1.00}$	s(0.00%)p(99.95%)d(0.04%)
π∗C2–C3	0.3354	$sp^{1.00}$	s(0.00%)p(99.96%)d(0.04%)
π∗C4–C5	0.3514	$sp^{1.00}$	s(0.00%)p(99.95%)d(0.04%)

The second-order perturbation energies (also known as the stabilization energy or interaction energy) of the most interacting NBOs of the studied molecules is presented in Table 11. The second-order perturbation energies consistent with the intramolecular hyper-conjugative interactions of 3,6-dibromo-p-xylene, 3,6-dichloro-p-xylene, 3,6-difluoro-p-xylene and P-xylene respectively which result into intermolecular charge transfer (ICT) causing stabilization of the systems respectively are presented in Tables S6, S7, and S8 of supporting information in detail**.** The most significant intramolecular hyperconjugative interactions which results in the highest stabilization energy of 206.98 kcal/mol, 20.53 kcal/mol, 20.52 kcal/mol, 20.56 kcal/mol, were obtained for π∗(C2–C3) →π∗(C4–C5), π(C4–C5) →π∗(C1–C6), π(C4–C5) → π∗(C2–C3), and π(C1–C6) → π∗(C4–C5) of DBPX respectively while 296.2 kcal/mol, 201.23 kcal/mol 20.53 kcal/mol, 20.44 kcal/mol were obtained for π∗(C3–C4) → ∗π(C1–C2), π∗(C5–C6) →σ∗(C1–C2), π(C1–C2) →π∗(C3–C4), and π(C3–C4) →π∗(C1–C2) for DCPX respectively and 21,44 kcal/mol, 21.08 kcal/mol, 20.54 kcal/mol and 19.94 kcal/mol were obtained for π(C1–C2) →π∗(C3–C4), π(C1–C2) →π∗(C5–C6), π(C3–C4) →π∗(C1–C2), and π(C5–C6) →π∗(C1–C2) of DFPX respectively. For p-xylene, the greatest interactions with the highest stabilization of 20.75 kcal/mol, 20.29 kcal/mol, and 20.19 kcal/mol were obtained for π(C1–C6) →π∗(C4–C5), π(C2–C3) →π∗(C1–C6), and π(C1–C6) →π∗(C2–C3) respectively. These strong interactions within the ring system as observed in the results suggest an intensely delocalized structure, the extra stability as observed for the fluorine, chlorine and bromine substituted isomers is due to resonance stabilization. That is, the stability is attributed to the backflow of electrons from the halogen lone pair into the aromatic ring by π-conjugation. This results show that the stability of the studied compounds with respect to the stabilization energy is in the order 3,6-dichloro-p-xylene > 3,6-dibromo-p-xylene > 3,6-difluoro-p-xylene > p-xylene i.e. it decreases as the reactivity and electronegativity value increases. The chlorine substituted derivatives is the most stable as observed due to multiple bond formation involving d-orbitals of the chlorine atom while the fluoro-substituted p-xylene derivative has the least stability as observed from the E(2) energy due to the increasing polarity of the C–F bond. The stability of halogens generally increases down the group in the periodic table and this result seems to correlate well. The entire trend observed can be attributed to the electronegativity and the negative inductive effect of the halogen atoms attached to the xylene ring. However, the stabilization energy only cannot give us a convincing proof with regards to the trend observed, therefore more experimental evidence is still needed to verify the order of stability observed.

**Table 11:** Second Order Perturbation Theory Analysis of the most interacting NBOs of the studied molecules using B3LYP/6-311+G functional. (^a^$\;E^{2}$ represent the energy of hyperconjugative interaction (stabilization energy). ^b^Energy difference between donor and acceptor E (i) and E (j) NBO orbitals. c F(i, j) is the Fock matrix element between i and j NBO. LP(n)A is a valence lone pair orbital (n) on atom A).

Most interacting NBOs for DBPX						
Donor	Occupancy	Acceptor	Occupancy	$E^{\left(2\right)a}$[Kcal/mol]	$E\left(j\right)-E{\left(i\right)}^{b}$[a.u.]	$F{\left(i,j\right)}^{c}$[a.u.]
σC1-C2	1.95508	σ∗C6–Br18	0.03687	6.03	0.79	0.062
πC1-C6	1.66232	π∗C4–C5	0.34300	20.57	0.30	0.070
		π∗C2–C3	0.38921	19.23	0.28	0.067
πC3-C4	1.69505	π∗C4–C5	0.34300	19.92	0.30	0.070
		π∗C1–C6	0.40658	18.83	0.29	0.068
πC4-C5	1.98006	π∗C1–C6	0.40658	20.53	0.27	0.068
		σ∗C2–C3	0.02309	20.52	0.27	0.067
π∗C2–C3	0.38921	π∗C4–C5	0.34300	209.98	0.01	0.083
LP(3) Br17	1.93740	π∗C2–C3	0.38921	9.27	0.31	0.052
LP(3) Br18	1.93740	π∗C1–C6	0.40658	9.30	0.31	0.053
DCPX						
σC1-C2	1.95874	σ∗C3–Cl18	0.03310	5.43	0.84	0.060
πC1-C2	1.65267	π∗C3–C4	0.41016	20.53	0.27	0.068
		π∗C5–C6	0.39388	20.33	0.27	0.067
πC3-C4	1.66032	π∗C1–C2	0.34553	20.44	0.30	0.070
		π∗C5–C6	0.39388	19.43	0.28	0.067
πC5-C6	1.69334	π∗C1–C2	0.34553	19.73	0.30	0.070
		π∗C3–C4	0.41016	19.14	0.29	0.068
LP(3)-Cl17	1.93026	π∗C5–C6	0.39388	11.73	0.34	0.061
LP(3)-Cl18	1.93026	π∗C3–C4	0.41016	11.73	0.34	0.061
π∗C3–C4	0.41016	π∗C1–C2	0.34553	296.23	0.01	0.080
π∗C5–C6	0.39388	σ∗C1–C2	0.03593	201.23	0.02	0.083
DFPX						
πC1-C2	1.67649	π∗C3–C4	0.39138	21.44	0.28	0.071
		π∗C5–C6	0.37884	21.08	0.28	0.069
πC3-C4	1.64731	π∗C1–C2	0.37779	20.54	0.29	0.070
		π∗C5–C6	0.37884	19.71	0.29	0.067
πC5-C6	1.68153	π∗C1–C2	0.37779	19.94	0.30	0.070
		π∗C3–C4	0.39138	19.48	0.30	0.069
LP(3)-F17	1.93214	π∗C3–C4	0.39138	16.58	0.44	0.083
LP(3)-F18	1.93214	π∗C5–C6	0.37884	17.05	0.43	0.083
PX						
πC1-C6	1.6496	π∗C4–C5	0.3514	20.75	0.28	0.069
		π∗C2–C3	0.3354	20.19	0.28	0.067
πC2-C3	1.6797	π∗C1–C6	0.3514	20.29	0.29	0.069
		π∗C4–C5	0.3514	20.29	0.29	0.069
πC4-C5	1.64961	π∗C1–C6	0.3514	20.75	0.28	0.069
		π∗C2–C3	0.3354	20.19	0.28	0.067

From the NBO analysis results, it can be inferred that despite fluorine being the most electronegative of the halogens, it is seen to be the most activating of the studied substituted halogen. This activation can be attributed to the better orbital overlap of the fluorine 2p orbitals with the p orbitals of the pi-system which results in a stronger pi-bond [31]. This can be confirmed by comparing the stabilization energies of the non-bonding interactions of the studied halogen the LP(3) F17 →π∗(C3–C4) and LP(3) F18→π∗(C5–C6) is seen to give the strongest stabilization of 16.58 kcal/mol and 17.05 kcal/mol respectively while the LP(3) Cl17 →π∗(C5–C6) and LP(3) Cl18→π∗(C3–C4) is seen to give the stabilization energy of 11.73 kcal/mol each respectively whereas the bromine halogens is seen to give the lowest non-bonding interaction corresponding to LP(3) Br17 →π∗C2–C3 and LP(3) Br18 →π∗(C1–C6) with the stabilization energy of 9.27 kcal/mol and 9.30 kcal/mol respectively. the higher the stabilization energy of the non-bonding interactions, the stronger the backflow of electrons from the halogen lone pair into the aromatic ring and the stronger the interaction. Fluorine is seen to have the highest non-bonding interaction which makes it a better pi-donor. These stabilization interactions between the lone pair orbitals and the anti-bonding orbitals account for the biological activity of these molecules. This results also confirms the assertion from literature [31] that the halogen atom confers both negative inductive effect and positive resonance effect on the benzene ring and the overall effect is electron-withdrawing. This effect can be seen from the stabilization energies reported above, that Chloro and Bromo p-xylene give a high stabilization energy corresponding to pi to pi∗ C–C bond on the aromatic ring thus conferring stability by resonance but the electron-withdrawing effect of the fluorine atom is seen to cause a decrease in energy in those pi-transitions but with an increase in the LP to π∗ interaction energy. The stability of the Fluoro, Chloro, and Bromo-p-xylene is seen to be more compared to that for para-xylene as a result of the strong interaction and co-planarity of the halogen substituent with the ring which enhances the electron delocalization from the halogen to the aromatic ring and back from the aromatic ring to the halogen atoms. This results seem to be in line with some other results reported in previous literature; Venkatesh *et. al.* [1] reported the structural and optical properties of 2,5-dichloro-p-xylene using DFT and observed from the NBO analysis two types of chlorine antibonding (Cl9 and Cl10) with their respective stabilization energy of 12.45 kcal/mol and 11.68 kcal/mol corresponding to Cl9 (LP) →π∗(C2–C3) and Cl10 (LP) →σ∗(C1–C2) respectively. In the interim, we also observed two types of chlorine antibonding (Cl17 and Cl18) with stabilization energy as reported in Table 11. This strong interactions around the ring could enhance the bioactivity of 2,5-dichloro-p-xylene. Jeyavijayan *et al.* [32] also reported the vibrational spectra, DFT calculations, electronic and optical properties of 3-bromo-o-xylene and confirmed from the NBO analysis that the pharmaceutical and biological properties of 3-bromo-o-xylene depends on the charge transfer evidence in the n3(Br15) →π∗(C1–C6), n2(Br15) →π∗(C2–C3), π(C2–C3) →π∗(C4–C5) etc. transitions with an interaction energy of 9.55, 3.34 and 19.88 kJ/mol respectively. This work has also noted the strong interaction between the halogen atom and the aromatic ring as reported in supporting information Tables S6, S7, and S8 and as, such affirms that the halogen atoms present in the xylene system confer some biological activity and stability to the para-xylene molecule.

### 3.6 Quantum chemical descriptors

The quantum mechanical descriptors using B3LYP/6-3211G functional are HOMO, LUMO, energy gap, electron affinity (EA), ionization potential (IP), hardness, softness, electronegativity, and electrophilicity index (ɯ) [24] as presented in the supporting information. The quantum chemical descriptors are quantitatively explained by considering Koopman's theorem [16].

$$\text{IP}=-E_{HOMO}$$

$$\text{EA}=-E_{LUMO}$$

Using Koopman's theorem for closed shell molecules (η), (σ), (X) can be redefined as;

$$\text{X}=\frac{IP+EA}{2}=-\mu ;\;\eta =\frac{IP-EA}{2};\;\sigma =\frac{1}{\eta };$$

The electrophilicity index(ɯ) formula is ɯ$=\frac{\mu^{2}}{2\eta }$

In the simplest terms, the hardness of a species, atom, ion, or molecule, is a qualitative indication of how polarizable it is, that is, how much its electron cloud is distorted in an electric field. The hard and soft concept proved useful, particularly in rationalizing acid-based chemistry [33, 34]. Hard and Soft Acids and bases [35]. So the chemical hardness and softness of a molecule is a measure of the stability of the molecule. Molecules having a low value of the energy gap are referred to as soft molecules (there are more polarizable), whereas molecules having high energy gap are called hard molecules. According to Janak [36,37] theorems, MO theory approaches, the HOMO energy is directly related to the IP, while the LUMO energy has been used to estimate the electron affinity (EA), making it possible to calculate other quantum chemical descriptors such as electron affinity, ionization potential, hardness, softness, electronegativity, and electrophilicity index.

From the results, the compound which has the lowest energy gap is DBPX. Therefore, this lower energy gap allows it to be the softest molecule. Also from our analysis, the compound that has the highest energy gap is PX. Which shows it is the hardest molecule. The compound that has the highest HOMO energy is PX. This implies that PX is the best electron donor. While the compound that has the lowest LUMO energy is DBPX which signifies it is the best electron acceptor. PX has the lowest value of ionization energy, thus it is a better electron donor this further confirms its highest HOMO energy. DBPX has the largest value of electron affinity indicating that it is the better electron acceptor which also confirms the idea of it having the lowest LUMO energy.

The chemical hardness of DBPX is the least among all the molecules. Thus, it is the most reactive among all the molecules, and therefore, reactivity decreases in the order DBPX > DCPX > DFPX > PX. This trend however is based on the concept of hardness and softness which only might not offer complete and convincing evident for the reactivity of the compounds is question. The highest electrophilicity index value of DCPX indicates that it is the strongest electrophile of all the compounds. It is observed that the value of and other quantum mechanical descriptors for 3,6 DCPX using B3LYP/6-311+G basis set is close to that observed from the experimental and theoretical study of the structural, electronic and optical properties of 2,5DCPX [1].

## 4 Conclusion

The basic chemistry of p-xylene, 3,6-dibromo-p-xylene, 3,6-dichloro-p-xylene and 3,6-difloro-p-xylene in terms of reactivity, stability and interaction have been discussed in this study extensively. Optimization of this compounds was done with GAUSSIAN 09 of density functional theory (DFT) method of B3LYP/6-311+G(d,p) basis set. Vibrational energy distribution analysis (VEDA) 04 and natural bond orbital (NBO) 7.0 were used for the analysis. The studied compounds are said to show biological activities. And the intramolecular hyperconjugative interactions responsible for stabilizing the compounds have also been identified. The NBO results also revealed that the non-bonding interaction existing between the lone pair electron on the halogen atoms and the aromatic ring increases the stability of the halogen substituted para-xylene molecules. The studied compounds were observed to show increasing stability and decreasing reactivity moving from DBPX, DCPX, DFPX to PX as shown from the observed HOMO-LUMO values. The Raman spectra of the studied compounds are also found in the supporting information. This research only gives a theoretical perspective of the stability and reactivity of p-xylene derivatives, however, more experimental research is still needed to validate the assertions made in this study and as such we recommend that further experimental and theoretical methods with greater accuracy should be employed to further understand the stability and reactivity of the studied compounds.

## Declarations

### Author contribution statement

Emmanuel A. Bisong, Hitler Louis: Conceived and designed the experiments; Performed the experiments; Analyzed and interpreted the data; Wrote the paper.

Tomsmith O. Unimuke, Joseph O. Odey, Emmanuel I. Ubana, Moses M. Edim, Fidelis Timothy Tizhe: Performed the experiments; Analyzed and interpreted the data; Wrote the paper.

Patrick M. Utsu: Contributed reagents, materials, analysis tools or data; Wrote the paper.

### Funding statement

This research did not receive any specific grant from funding agencies in the public, commercial, or not-for-profit sectors.

### Data availability statement

Data will be made available on request.

### Declaration of interests statement

The authors declare no conflict of interest.

### Additional information

No additional information is available for this paper.

## Appendix A Supplementary data

RE-2-REVISED MANUSCRIPT ON P-XYLENE. DFT STUDY RE-2-REVISED MANUSCRIPT ON P-XYLENE. DFT STUDY
